# Intelligent Measurement and Analysis of Sewage Treatment Parameters based on Fuzzy Neural Algorithm with ARM9 Core CPU

**DOI:** 10.1155/2022/3498060

**Published:** 2022-07-18

**Authors:** Yaqi Ma

**Affiliations:** School of Transportation, Soochow University, Suzhou 333403, China

## Abstract

After entering the new century, the state continues to increase the construction of urban sewage treatment projects in response to the deteriorating water pollution situation. How to collect and analyze the sewage parameter variables in the sewage treatment process to ensure the intelligent measurement and accurate operation of the parameters in the treatment application is an urgent problem to be solved. This paper is mainly based on the computer-aided control system built by the ARM9 core embedded chip, and the feasibility and effectiveness of fuzzy neural network algorithms are discussed to improve the intelligent processing of sewage treatment parameters. After analyzing the principle and implementation flow of fuzzy control and neural network, starting from the characteristics of data collected by ARM9 core chip, the hybrid algorithm model is optimized and improved to further improve the convergence speed and accuracy of the algorithm. The simulation experiment proves that the optimized fuzzy neural control algorithm can effectively identify the dissolved oxygen, nitrate nitrogen, and other parameter data in the sewage treatment, and the recognition accuracy is very close to the true precision. Based on biosensors, the ARM9 core chip control system established by a recursive fuzzy neural network can greatly improve the tracking and control ability of parameters such as dissolved oxygen concentration and nitrate nitrogen concentration in microbial degradation. This has a good development prospect in wastewater treatment control applications. The experimental results show that the recursive fuzzy neural network algorithm proposed in this paper can dynamically track and control the nitrate concentration and dissolved oxygen concentration and ensure that the control is within the accuracy range. The accuracy of recognition is very close to the real accuracy.

## 1. Introduction

With the advent of the digital age of information technology in the field of water pollution control, the traditional use of manual treatment of sewage treatment information has been ended. This not only requires a lot of manpower and material resources and time but also has low precision and cannot meet the needs of today's digital construction and intelligent control. In this development background, the computer-aided control system based on the ARM9 core embedded chip uses intelligent sensor technology to collect real data in sewage treatment and takes advantage of the low energy consumption and high cost performance of the ARM9 embedded microprocessor, using the computer CPU. The comprehensive data operation analysis capability can effectively improve the intelligent level of sewage treatment. The ARM9 processor can perform sensor data acquisition in the automatic running state of the computer system. In order to reduce the error value between the sampled value and the set value, the fuzzy neural network algorithm can be used to control the ARM9 actuator. The sensor output signal is digitally filtered to remove interference through software and hardware, or the component measurement control can effectively improve the accuracy of the parameter measurement control.

Fuzzy control technology is a new type of strategy technology that simulates human reasoning ability and comprehensive analysis in the decision-making process. It is a representative application of machine intelligence control technology, which is mainly to solve the mathematical control model under nonlinear, multivariate, and factor conditions, which can effectively improve the adaptability, effectiveness, and rationality of traditional control algorithms. The principle of this technology can well simulate the control methods of workers with rich operational experience in wastewater treatment. Therefore, the fuzzy neural network algorithm is introduced in this paper to accurately and effectively analyze the parameters of ARM9 processor components in wastewater treatment. The main innovation is to improve the reliability and stability of the collected data from the characteristics of the dynamic relationship system of sewage treatment. The mathematical model of wastewater treatment is established by a recursive fuzzy neural network to simulate the change of parameter variables in wastewater treatment and provide accurate information on wastewater treatment for the ARM9 treatment controller to improve the accuracy of decision control.

This paper discusses four methods to improve the structure of a fuzzy neural network. The optimization of the fuzzy neural network algorithm is being studied. The innovative contributions include: combined with the analysis of the characteristics of the fuzzy neural network algorithm and the of sewage treatment data information, the fuzzy neural network algorithm is used to control the uncertain parameters. The influence of the algorithm learning rate on algorithm efficiency is studied. The effect and quality of the recursive fuzzy neural network algorithm are improved, and the adaptive change method is introduced for optimization, so that the network can achieve faster convergence while ensuring performance, so as to effectively improve the control response speed and accuracy. These fuzzy neural network algorithms effectively improve the application effect of the ARM9 processor in practical sewage treatment.

The structure of this paper is divided into five sections: the first section discusses the advantages of fuzzy neural network algorithms in ARM9 processor information analysis. The fuzzy neural network algorithm supported by computer-aided technology can study the analysis and processing of data faster and more effectively. The second section introduces the principle and advantages of the fuzzy neural network algorithm, puts forward the original intention of this paper, and analyzes the main principles and implementation process of the fuzzy neural network algorithm. The third section gives the design flow of the fuzzy neural network algorithm. In order to improve the accuracy and reliability of the existing fuzzy neural network algorithm, an optimization strategy is proposed. In the fourth section, the optimization strategy of the fuzzy neural network algorithm is proposed, and the performance characteristics of the optimized fuzzy neural network algorithm are introduced. The fifth section summarizes the research content of optimizing fuzzy neural network algorithms and analyzes the development direction of the ARM9 processor and computer-aided technology in the field of sewage treatment data control.

## 2. Related Work

Many scholars have conducted multi-level and multi-angle research on wastewater treatment technology based on computer-aided technology. Baawain et al. proposed a decentralized prediction model to study the hydrogen sulfide emissions in wastewater pollutants and discussed the feasibility and effectiveness of total control modeling for wastewater prediction research [1]. Qiu et al. proposed to use biofilm to realize the automatic control system in the secondary water treatment by studying the decentralized wastewater of Tianjin Modern Agricultural Science and Technology Innovation Base. The simulation experiment proved that the research could effectively purify the decentralized wastewater [2]. Based on the characteristics of the sewage treatment process, Hong et al. proposed a controller parameter adjustment strategy based on the BP neural network. The experiment proved that the dissolved oxygen concentration in wastewater treatment had better control precision and effect than the traditional controller [3]. Tang et al. explored the treatment strategy for constructed wetland wastewater, explored the use of ecological control systems to improve the environmental protection of wastewater, and used the effects of mixed strains to comprehensively control the growth of strains to achieve environmental protection of wetlands [4]. Kühr et al. explored how current wastewater treatment plants could use engineering nanoparticles to improve the effect of wastewater treatment. The comparative experiments showed that engineering nanoparticles could play a very good role in inducing ecotoxicological effects, and the application space was very broad [5]. Giang et al. studied the carp that survived the wastewater treatment plant's wastewater pool and explored the effects of sewage treatment on the organism. The study concluded that the wastewater from the wastewater treatment plant would have many negative impacts on the development of the organism and needs to be highly valued [6]. Krishna Reddy et al. studied urban sewage treatment technology in a cold environment and proposed an improved sewage treatment system. They improved denitrification efficiency to improve nitrogen treatment in wastewater and heated exchangers to increase ambient temperature to improve treatment efficiency [7]. After studying the wastewater composition of developing countries in South Africa, Oberholster et al. explored strategies for improving wastewater treatment efficiency in terms of urban household wastewater and wastewater treatment in rural areas [8]. Tang et al. mainly conducted research on the treatment of drugs in two major sewage treatment plants in Guangdong Province. It was found that most drugs were seasonalized by stratification of the target drugs such as clofibrate and ibuprofen in the front and back of sewage treatment. The impact of the change the overall removal of the drug from the sewage plant would be subject to changes in the concentration of seasons and time [9].

The application research of fuzzy control technology by domestic and foreign scholars was more in-depth and extensive, and there were also many research results worthy of reference in fuzzy neural network algorithms. Zhangwen et al. studied the feasibility of applying fuzzy control technology to wavefront correction. It was believed that the technical department was subject to the response model of the deformable mirror, and the wave front correction effect required by the adaptive engineering system could be realized by evaluating the fuzzy proportional integral differential control. Experiments showed that the technique could achieve good control effects and accuracy [10]. Heng et al. mainly discussed the use of fuzzy control technology to improve the output accuracy of the missile's inertial component unit in the dynamic environment. It was proposed to automatically adjust the stiffness and damping of the self-retaining elastic body by changing the magnetic field to achieve the vibration response efficiency of the inertial measurement unit. The output accuracy has improved [11]. Wang et al. explored the use of fuzzy partial differential equations to learn the stability of spatially sampled data. It was proposed to use the fuzzy controller with data to accurately confuse the complex spatiotemporal dynamics of nonlinear fuzzy partial differential equations. Simulation experiments showed that this method improved the performance of data fuzzy controllers [12]. ZhongZhong used an event-based strategy to design a distributed controller to solve the stability problem of the microgrid. A certain number of PV arrays are combined into a buck converter, and the structural design of the distributed controller is improved based on the event. The scheme can also ensure the stability of the microgrid in the case of fewer communication resources [13]. Tang et al. used fuzzy neural networks to construct a prediction model of vehicle speed in long-distance traffic. Based on the fuzzy inference principle, the two learning processes based on fuzzy neural networks effectively improved the accuracy of the prediction model and reduced the error rate of prediction [14]. Qiao et al. proposed a second-order self-organizing fuzzy neural network to predict the concentration of fine particles in the air in China. In order to improve the sensitivity of the model output, a two-step algorithm was applied to learn the parameters, thereby improving the prediction accuracy of the final hybrid model. Experiments show that the model has satisfactory prediction results [15].

Through scholars' research on the performance of the ARM9 embedded microprocessor under computer-aided technology, fuzzy intelligent control technology, and fuzzy neural network algorithms, it can be seen that artificial intelligence algorithms take advantage of computer data processing in the field of sewage treatment, which can effectively improve the level of intelligent control in many industries. Therefore, this paper mainly focuses on the fuzzy neural network algorithm to control the parameter data of the ARM9 processor.

## 3. Methodology

### 3.1. Fuzzy Control and Neural Network Algorithm

Ambiguity refers to something that has no exact meaning in essence, has no clear indicators in quantity, and has an unclear state at the boundary. It is an excessive phase between things that have obvious differences. The basis for the ambiguity of things is fuzzy mathematics. Fuzzy set theory is to study unclear and uncertain fuzzy things with clear and clear mathematical methods, which is the link between fuzzy cognition and precise mathematical models [16]. In the late 1970s, Zadeh proposed the possibility theory. The technology based on fuzzy set theory and fuzzy logic is collectively called fuzzy technology, which is a process of simulating human thoughts and cognitions of fuzzy things. Fuzzy control is a kind of control of nonlinear parameters, which belongs to the field of machine intelligence control. This control method does not require the construction of an accurate mathematical model, and has the characteristics of simple operation and high reliability for process control of complex systems with many input parameters, large parameter denaturation and high nonlinear uncertainty [17].

As the core component of fuzzy control, a fuzzy controller has four characteristics. One is to convert a signal with a relatively accurate input into a corresponding set of fuzzy quantities. Second, the knowledge base of fuzzy control is composed of fuzzy language as the control rule represented by variables, which is the embodiment of specific operational experience and knowledge [18]. Third, fuzzy reasoning allows fuzzy control to simulate human thinking methods and can perform rule reasoning based on the association of fuzzy logic. Fourth, fuzzy control also has the ability to defuzzify and can convert the fuzzy variables obtained by fuzzy derivation to the actual operational variables that can be accurately controlled.  Figure 1 is a schematic diagram of a conventional fuzzy controller. There are two main types of rules for fuzzy control [19]. The first is the state evaluation fuzzy control rule, as shown in formula (1), which is a control method very similar to human intuition. The second is the target evaluation fuzzy control rule, which is the type of rule used to make predictions as shown in the following formula:

(1) $$\begin{array}{c} Ri:if\;x1\;is\;Azi1\text{ and }x2\;is\;Azi2\cdots \text{and }x\;is\;Ain \end{array}$$

(2) $$\begin{array}{c} Ri:if⟶\left(x\text{ is}A1y\;s\;B1\right)\text{then}U\;is\;Ci. \end{array}$$

The neural network is an information-feedforward layered neural network with typical characteristics of backward propagation. It is bidirectional propagation in the learning algorithm. Its network structure is divided into input layers [20], an output layer, and a hidden layer. The hidden layer here may be one layer or multiple layers, and each layer is forwardly linked by the connection weight between nodes. After a signal is input, the signal is transmitted to the hidden layer. After the excitation function is calculated, the information is transmitted to the output layer and changes to the output signal. The neural network training algorithm process is characterized by both forward and reverse propagation. When the signal adopts the “input layer-implicit layer-output layer” process, it reflects the state of forward propagation [21]. When the hidden layer receives the signal and produces an error with the output signal, and the error exceeds a desired range. Based on this error, the system will correct the weights and thresholds of each layer of neurons so that they become more adaptive to each other to promote system performance. This reacts to the state of back propagation. A single node in the network represents a neuron, and there is no connection between neurons in the same layer. The nodes of each layer only accept the input of the nodes of the previous layer, and the output of each layer of neurons only affects the nodes of the subsequent output layer. In practical applications, only one layer of the hidden layer can meet the needs of use [22]. When the hidden layer reaches three layers, it can reflect the mapping of any continuous function. The BP neural network is the most typical type of neural network, and its model structure is shown in Figure 2.

The BP neural network uses a learning algorithm with a tutor. The basic learning steps are: (1) Initializing the weights *w* and *θ*, the connection weight of the input layer to the hidden layer neurons is *w*_*ij*_. The connection weight of the hidden layer to the output layer is *w*_*jk*_. The threshold of the hidden layer is set to *θ*_*j*_. The threshold value *θ*_*k*_ of the output layer neurons is assigned a smaller value between (0, 1). (2) Determine the input vector *x*_*i*_=(*x*_1_, *x*_2_,…, *x*_*m*_) and the expected output vector $\overset{\wedge }{Y}=\left(\overset{\wedge }{Y_{1}},\overset{\wedge }{Y_{2}},\ldots ,\overset{\wedge }{Y_{n}}\right)$ corresponding thereto, input the value of *x*_*i*_ to the neuron node of the input layer, perform forward calculation according to *x*_*j*_^*i*^=*f*(∑_*i*=0_^*n*^*W*_*ij*_*x*_*i*_ − *θ*_*j*_)(*j*=1,2,…, *u*), or perform reverse calculation, for example, *y*_*k*_=*f*(∑_*k*=0_^*n*^*V*_*ij*_*x*_*j*_ − *θ*_*k*_)(*k*=1,2,…, *n*). The error between the output layer neuron output value and the expected output value is calculated. If the error result is in line with expectations, the training is over. If the gap is too large, it will enter the reverse calculation of the model calculation again.  Figure 3 shows the BP neural network learning algorithm flow.

### 3.2. Fuzzy Control and Neural Network Algorithm Optimization Strategy

The control of the sewage treatment process is a complex, dynamic relationship system. The stability and reliability of the system are important assessment indicators in practical applications [23]. Therefore, it is necessary to accurately grasp the various parameters information in the sewage treatment process through mathematical models, providing an important basis for the smooth control of the system. The number of fuzzy rules is the key to determining the performance and efficiency of the entire fuzzy neural network. In the case of too many fuzzy rules, the generalization ability of the neural network structure is reduced, and the training samples are over-fitting; when the network structure is increased, the network learning speed is reduced. If the fuzzy rules are too small, the learning ability of the neural network will deteriorate and the accuracy will not be enough [24]. Therefore, the current fuzzy neural network is mainly based on the structural optimization of the algorithm model. In this context, this paper establishes a mathematical model of wastewater treatment through a recursive fuzzy neural network to simulate the variation of parameter variables in wastewater treatment and provides a fuzzy controller with accurate information for wastewater treatment for decision control. The typical topology of a recursive fuzzy neural network is shown in Figure 4.

There are four main types of algorithms for the structural optimization of fuzzy neural networks. The first is the test-in method. The practical applicability of this method is relatively good. For different problems, it is necessary to construct different neural networks for training through the prior knowledge structure, and then proceed to the actual output, network output, generalization ability, structurality, etc. The best model is evaluated and found among them. This method is cumbersome and easy to enter the local values of the training, so it is very likely that the optimal model cannot be found. The second is the construction method, which is to make the neural network first small in size. In the training process, based on the needs of the network, the network weight and nodes are added to meet the network performance growth needs. The third is the destructive method, which is a construction method of the reverse principle of the construction method. The network being constructed first needs to be large in scale and have many nodes. In the training process, subtraction is used to remove unnecessary weights and nodes, and the complexity of the network is reduced. This way, when the generalization ability is enhanced, you can build the most streamlined network structure that satisfies performance. The fourth is evolutionary algorithms, such as the use of evolutionary strategies and genetic algorithms, through the joint model of algorithms and neural networks to achieve the best search for the global. Such models tend to be more stable.  Figure 5 is a schematic structure of a sewage treatment control system based on a fuzzy neural network.

Learning rate is a factor that has a direct impact on neural network learning. If the learner is too low, the learning process of the whole neural network will be too slow, and the learning rate will be too high, which will cause the network to be unstable and make the network learning unreliable. To solve this problem, an adaptive change method is introduced to optimize the stability and reliability of the entire neural network. The adaptive learning rate approach allows the network to achieve faster convergence while maintaining performance. The Lyapunov function is shown in the following equation . As shown in the following equation, at Δ*V* ≤ 0, the stability of the Lyapunov function can be guaranteed.

(3) $$\begin{array}{c} V\left(t\right)=J\left(t\right)=\frac{1}{2}\sum_{p=1}^{N0}e_{p}^{2}, \end{array}$$

(4) $$\begin{array}{c} \Delta V\left(t\right)=\Delta V_{1}\left(t\right)+\Delta V_{2}\left(t\right)+\cdots +\Delta V_{No}\left(t\right), \end{array}$$

### 3.3. Task Management of Sewage Treatment System

The system starts running, and the embedded operating system schedules each task. After the system is started, tasks are first established according to priority, and their priorities are allocated reasonably. *μ* Cos-II is responsible for the scheduling and synchronization of each task, and data sharing between each task is carried out through semaphore, mailbox message queue, and other communication mechanisms. The functions that the system needs to realize may be divided into two parts: first, complete the collection and storage of liquid level value, do, and COD data. Data acquisition uses the clock interrupt provided by pc/os-II to collect the liquid level value according to the time interval set by the system. Values of do, BOD, and COD sensors. Then the workload of the water pump group, aerator, and dosing device is determined according to the fuzzy algorithm. The task of sludge discharge is to use the clock interrupt provided by c/os-ii to control task of sludge discharge is to utilize *μ*. The clock interrupt provided by c/os-II is used for control. When the set time is reached, start the task of sludge discharge. The sludge discharge time is determined according to the operation experience of the sewage treatment plant. Secondly, the LCD touch screen displays the communication between human-machine interface tasks. Parameter setting, display of collected data, receiving commands, and performing tasks were performed as required.

The human-computer interface task has the highest priority, and each task is created first in the human-computer interface task. Then start the task. The first task to be called and executed is the LCD touch screen display task. In LCD display and touch tasks, first set parameters such as liquid level warning value and sludge discharge time. After parameter setting, it will wait for system messages sent by other tasks. Then the corresponding operations are performed according to the received message priority, and the task is in a continuous waiting state. The ready state cannot be reached until a message enters the message queue. After the human-computer interface task is suspended, the data acquisition task enters the running state. In this task, the program reads the measured object data from the processor's AD conversion register. By comparing the data with the preset value, the fuzzy control algorithm is used to determine the pump workload of the sewage treatment pump house, the aeration of the aeration tank, the dosing of the sedimentation tank, and other parameters.

## 4. Optimize the Performance Experiment of Fuzzy Neural Network Algorithm

### 4.1. Experimental Conditions and Parameters

In order to verify the parameter control performance of the recursive fuzzy neural network algorithm introduced in this paper, the simulation experiment was carried out. The experimental data is derived from M Company, which uses industrial benzene as its main raw material. The company produces chemical products such as rubber auxiliaries based on various anilines. The wastewater produced during the production process is mainly used for washing wastewater in product separation and fine processes. The benzene and phenolic pollutants contained in the wastewater have higher indexes. The company uses biosensor-based microbial purification processes for the biochemical treatment of wastewater.

The simulation experiment is based on a computer-aided platform, and the experimental data is collected in a 20-day cycle in wastewater treatment. The data of the previous 10 days is used as the training sample of the neural network, and the data of the following ten days is used as the test sample of the network to compare and verify the data. The computer environment in the experiment is the Linux operating system, in which the CPU module circuit uses the microprocessor of the Samsung ARM9 core. The fuzzy neural network is used to realize the intelligent adjustment of the parameters of each link of the embedded control system.

### 4.2. Algorithm Performance Experiment

The recurrent neural network was proposed in 1990 and is regarded as a generalization of the recurrent neural network. When each parent node of a recurrent neural network is connected with only one child node, its structure is equivalent to that of a fully connected cyclic neural network. Recurrent neural networks can introduce gated mechanism to learn long-distance dependence. Recurrent neural networks have flexible topology and weight sharing. It is suitable for machine learning tasks containing structural relationships. It has important applications in the field of natural language processing (NLP). In the experimental application, the online pollutants are identified in the form of online modeling. Here, the recursive fuzzy neural network is used to establish the controller. The input value of the controller is set. There is a certain allowable error between the input value and the actual output. In order to effectively test the control effect of the recursive fuzzy neural network proposed in this paper, the experiment uses the method of setting variables. The dissolved oxygen value is set to 1.9 mg/L for 11-12 days. The dissolved oxygen value was set to 2.3 mg/L in 13-14 days. The dissolved oxygen value is set to 1.3 mg/L for 15–20 days. On other days, the dissolved oxygen value is set to be fixed at 2 mg/L. The concentration of nitrate nitrogen in the period of 11-12 days is set at 0.9 mg/L. The concentration of nitrate nitrogen is set at 1.3 mg/L in 13-14 days. The concentration of nitrate nitrogen is set at 1.1 mg/L for 15–20 days. The simulated simulation results of the dissolved oxygen recognizer obtained in the experiment are shown in Figure 6.

Figure 7 shows the effect of the dissolved oxygen concentration control. As can be seen from the figure, although the experiment has different settings for the pre-values, the recursive fuzzy neural network recognizer can effectively identify the dissolved oxygen and nitrate nitrogen in the case of setting changes. Moreover, the accuracy of the recognition is very close to the true accuracy.

Figure 8 is a comparison of the effects of nitrate concentration control. It can be seen from the comparison of the above two control effects that the controller based on biosensor and recursive fuzzy neural network proposed in this paper can control the dissolved oxygen concentration and nitrate nitrogen concentration in microbial degradation. The range of errors is relatively small and has a good prospect of practical application.

As can be seen, the concentration of nitrate nitrogen is mainly controlled in sewage treatment control. The recursive fuzzy neural network algorithm proposed in this paper has a good advantage for the control efficiency, cycle, and execution time. Therefore, based on the optimized fuzzy control network algorithm proposed in this paper, the control effect of the ARM9 microprocessor can be effectively improved, and the tracking and control of dissolved oxygen concentration and nitrate nitrogen concentration in aniline wastewater treatment can be realized, and the control can be guaranteed within the accuracy range.

In the experimental application, on-line pollutants are identified in the form of on-line modeling. The recursive fuzzy neural network is used to establish the controller and set the input value of the controller. There is a certain allowable error between the input value and the actual output. The experiment adopts the method of setting variables. The control effect of the recurrent fuzzy neural network proposed in this paper is effectively tested. Recursive fuzzy neural network recognizer can effectively identify dissolved oxygen and nitrate nitrogen in the case of setting changes. In addition, the recognition accuracy is very close to the real accuracy. The controller based on biosensors and recurrent fuzzy neural networks can control the concentration of dissolved oxygen and nitrate nitrogen in the process of microbial degradation. Compared with traditional technology, embedded systems have the advantages of small size, low power consumption, strong specificity, and high real-time, which makes it favored by the majority of users since its emergence, and its development speed is very rapid. The emergence of some open-source operating systems has contributed to its global popularity. When it is applied to engineering practice, it will inevitably produce huge economic and social benefits, and its application prospects are very broad.

## 5. Conclusion

A fuzzy neural network is a mathematical model constructed by fuzzy theory and a neural network algorithm. It has the ability to solve nonlinear, multivariate, and multifactor conditions, and can effectively improve the adaptability, validity and rationality of traditional control algorithms. Therefore, the fuzzy neural network algorithm was introduced to control the parameters of the ARM9 microprocessor to improve the accuracy of related parameter management and control in the wastewater treatment process. Based on the analysis of the principle and implementation flow of fuzzy control and neural network algorithms, this paper proposes an optimization scheme for recursive fuzzy neural networks based on the dynamic complexity of system control for the needs of relevant parameters in wastewater treatment. The model is to accurately grasp the various parameter information in the wastewater treatment process to ensure the validity and reliability of the model, thus providing an important basis for the smooth control of the system. After that, simulation experiments were carried out on the treatment of aniline wastewater from M chemical companies. The experimental results show that the recursive fuzzy neural network algorithm proposed can dynamically track and control the nitrate concentration and dissolved oxygen concentration and ensure that the control is within the range of precision. The accuracy of recognition is very close to the true precision. From the verification results, there are still some improvements in this study. The next step is to conduct in-depth research at the execution time of the fuzzy neural network.

## Figures and Tables

**Figure 1:** The principle diagram of commonly used fuzzy controllers.

**Figure 2:** Structure of BP neural network.

**Figure 3:** Neural network BP learning algorithm flow chart.

**Figure 4:** Typical topology of recurrent fuzzy neural networks.

**Figure 5:** Principle structure of a wastewater treatment control system based on fuzzy neural network.

**Figure 6:** Modeling effect of dissolved oxygen identifier.

**Figure 7:** Control effect of dissolved oxygen concentration.

**Figure 8:** Control effect of nitrate nitrogen concentration.

## Data Availability

The data underlying the results presented in the study are available within the manuscript.
